# Cancer in Africa: Is It a Genetic or Environmental Health Problem?

**DOI:** 10.3389/fonc.2020.604214

**Published:** 2020-12-14

**Authors:** Abeer A. Bahnassy, Mona S. Abdellateif, Abdel-Rahman N. Zekri

**Affiliations:** ^1^ Tissue Culture and Cytogenetics Unit, Pathology Department, National Cancer Institute, Cairo University, Cairo, Egypt; ^2^ Medical Biochemistry and Molecular Biology, Cancer Biology Department, National Cancer Institute, Cairo University, Cairo, Egypt; ^3^ Molecular Virology and Immunology Unit, Cancer Biology Department, National Cancer Institute, Cairo University, Cairo, Egypt

**Keywords:** Africa, cancer, incidence, survival, mortality

## Abstract

Patients of African ancestry have the poorest outcome and the shortest survival rates from cancer globally. This could be attributed to many variables including racial, biological, socioeconomic and sociocultural factors (either single, multiple or combined), which may be responsible for this major health problem. We sought to assess the most common types of cancer that endanger the health of the African people, and tried to investigate the real differences between African and other Non-African patients regarding incidence, prevalence and mortality rates of different cancers. Therefore, identifying the underlying aetiological causes responsible for the increased incidence and mortality rates of African patients will allow for changing the current plans, to make optimized modalities for proper screening, diagnosis and treatment for those African patients, in order to improve their survival and outcomes.

## Introduction

Cancer is a major public health problem worldwide. It is one of the most leading causes of death in several regions depending upon disparities among different people (1). These disparities include socioeconomic, ethnic, racial and cultural factors that differ between low and high-income countries. According to the records obtained from the GLOBOCAN 2018 database of the International Agency for Research on Cancer (IARC) (2), the estimated results of 36 cancer types available from 47 countries of the African region of WHO (AFRO) revealed that there are 811,200 new cancer cases (4.5% of the total world) and 534,000 cancer deaths (7.3% of the total world) reported in the AFRO countries in 2018 (**Figure 1**).

**Figure 1:** The number of new cancer cases in AFRO region. **(A)** In African females, **(B)** in African males. Reproduced from “The Global Cancer Observatory, Africa Globocan 2018” (3).

The estimated cancer burden in the AFRO countries is mainly attributed to breast cancer which represents 27.7% of the total cancer cases, followed by cervical cancer which represented 19.6% of the total cases. Taken together, this represents the most common in African females. Meanwhile, prostate cancer (18.1% of total cases), followed by liver cancer (9.7% of total cases) and colorectal cancers (6.9% of total cases) were the most common in African males (**Figure 2**). Concerning survival rate of childhood malignancies, the survival rate is as low as 20% in African children and 80% in high income countries (4).

**Figure 2:** The top 10 cancers in African patients. **(A)** Age-standardized incidence rates per sex, **(B)** Age-standardized incidence and mortality rates. Reproduced from “The Global Cancer Observatory, Africa Globocan 2018” (3).

In an interesting study, Pinheiro and his colleagues (5), analysed the cancer mortality data obtained from South Florida for white, Hispanic, and black populations with disaggregation for Cuban, Puerto Rican, South American, African American, and Afro-Caribbean groups, during the period 2012–2016. Pinheiro et al., provided an evidence that, the African American males and females had the highest all sites-combined cancer mortality rates among all groups. As well as the highest mortality rates for many cancers including breast, prostate, lung, stomach, colorectal carcinoma, liver and multiple myeloma. According to their data, the Afro-Caribbean patients had significantly higher mortality rates compared to the white populations especially for stomach, prostate, multiple myeloma, premenopausal breast and endometrial carcinomas. In contrast, lower rates were reported for the other cancer types, particularly the lung cancer. These data are similar to other previous studies reported higher race-specific rates among both Afro-Caribbean and African American populations for endometrial, premenopausal breast, prostate, and multiple myeloma cancers in South Florida’s black population (6, 7). They also reported that lung cancer was the first leading cause of cancer-related death in African American men, followed by Prostate and colorectal cancers. While, for the Afro-Caribbean’s and other Hispanics, prostate cancer was the leading cause of cancer- related death followed by lung and colorectal carcinoma. On the other hand, breast and lung cancers were the first and the second leading causes of cancer- related death in African American females, followed by colorectal cancer, while lung cancer preceded breast and colorectal cancers in the Afro-Caribbeans (5).

It is a well-known fact that, cancer outcome is not equal in all people, and there are many factors that can affect its behaviour and its impact on the patients’ survival or response to treatment. Here, we review the most common types of cancer that endanger the health of the African people or those with African ancestry, and investigate the differences between African and non-African patients regarding incidence, prevalence, and mortality rates of different types of cancer. This will pave the way to produce an appropriate screening method or targeted therapy for such patients.

## Prostate Cancer

Prostate cancer is the first leading cause of cancer deaths in African males, and the second leading cause of cancer deaths in the united states (1, 2). It was obviously noted that, racial disparity plays a crucial role in its incidence and mortality rates among American patients (8). In 2007, It has been reported that prostate cancer incidence among black men in the US was 60% higher and its mortality was more than double the estimated rates in white men respectively (9). Later on, Siegel et al. (8), reported in 2014 that African-American men were 2.4 and 5.0 times more likely to die from prostate cancer compared to Americans of European or Asian ancestries, respectively. Various studies tried to investigate this racial disparity in prostate cancer regarding its incidence, prevalence, aggressive behaviour, and mortality rates. Some of these studies proposed that, the poor outcome in black men may be attributed partially to the inaccessible medical care and/or inadequate screening and treatment facilities (10, 11). Meanwhile, other studies mentioned the differences in germline and genetic background between black and white men as a reason (9, 12–14). Moreover, the socioeconomic status and lifestyle variation had also been suggested, however after adjusting for these factors, African ancestry remains a significant risk factor for prostate cancer (15). Supporting these data, Moul et al. and Faisal et al. (16, 17), concluded that the black race has to be considered an independent prognostic factor for disease recurrence, allowing for a more biologically aggressive phenotype. Though, the explanation of this disparity is still unknown and require more in depth studies (18). Tsodikov and his colleagues have also investigated this issue through establishing three predictive models of prostate-specific antigen (PSA) screening patterns in the USA, to compare the prostate cancer natural history in black men compared to the general population using an updated reconstruction of PSA screening. The obtained data were collected through the National Health Interview Survey in 2005, and the prostate cancer incidence from the Surveillance, Epidemiology, and End Results program (SEER) in 1975–2000 (18). They found that 30–43% of black men developed preclinical prostate cancer by the age of 85 years, which was relatively 28–56% higher than in the general population. Also, black men showed a similar risk of diagnosis (35–49%) compared to the general population (32–44%), but their risk of progression to a metastatic disease by the time of diagnosis was 44–75% higher than in the general population. Taken together, these results are consistent with those published by Powell et al. (19), which based on autopsy and surgical pathology data. They observed that black men have an increased risk of transformation to clinically significant cancer compared to white men.

Blackburn and his colleagues (20) tried to investigate the association between the underlying genetic differences for prostate cancer with the racial variations among peoples. They reported a lower frequency for *TMPRSS2‐ERG* fusion which is inversely associated with aggressive prostate cancer in black South Africans males compared to those from European ancestry. Similarly, Zhou et al. (21), performed a meta-analysis study and reported that the highest incidence of *TMPRSS2‐ERG* fusion was recorded in 49% in men of European ancestry. While, lower incidence rates were found in Asian (27%) and African (25%) male ancestries. Moreover, Magi-Galluzzi et al. (22) reported a racial discordance in the mechanism(s) of *TMPRSS2‐ERG* fusion occurrence, since the African Americans more commonly had *TMPRSS2‐ERG* fusion through deletion, whereas the European and Asian Americans had *TMPRSS2‐ERG* fusion through translocation.

For more confirmation of these data, an interesting study was done by Jaratlerdsiri et al. (23), who performed deep whole-genome sequencing for paired tumor-normal tissues obtained from African patients compared to non-African patients. The results of the study revealed a 1.8-fold increase in the small somatic variants, and also elevated oncogenic driver mutations in the African- derived tumors in comparison to the European counterpart. The *ERG* fusions and *PIK3CA* mutations were absent, *PTEN* loss was less frequent, whereas *CCND1* and *MYC* were frequently gained. In addition, out of the commonly affected prostate cancer gene pathways, genes regulating the calcium ion-ATPase signal transduction were disrupted in the African tumors. Therefore, it is quite clear that, a special screening program for the black men of African ancestry is highly required, and this should be done depending upon their own genetic makeup.

## Breast Cancer

Breast cancer (BC) is the most commonly diagnosed cancer in the African females, and it also represents the second leading cause of cancer- related deaths following cancer cervix in sub-Saharan Africa (SSA) (2). Its incidence had been increased in the last six years by more than 23% (from 1.7 million new patients in 2012 to 2.1 million in 2018) (24, 25). In addition, its five-year survival rate is less than 40% in SSA, compared to 86% in the United States (26). In their observational study on BC patients from USA, Iqbal et al. (27), reported that black women with small-sized tumors had 9.0% increase in the risk of death compared to the non-Hispanic white women who had only 4.6% increased risk of death. These data are in accordance with many previously published studies which showed that black women usually have higher risk of BC recurrence regardless of the age, tumor size or tumor grade. Based on these data, the African ancestry, by itself, should be considered an independent predictor factor for poor survival rates (28, 29).

Although BC mortality rate is now decreasing in the developed countries due to the implementation of screening programs including mammography, which is the gold standard for early detection and successful management of BC. The screening of BC in Africa is still a great challenge (30). This is attributed mainly to the lack of financial and technical support, in addition to decreased numbers of well-trained radiologists and technicians (31, 32). It was reported in some previous studies that, the age of peak incidence of BC is lower in SSA, with most of the women had advanced-stage disease at the time of diagnosis (33). At the same time, mammography is less effective for detecting tumors at advanced stages, as well as in younger women due to changes in breast tissue density according to the hormonal profile of the patients (34). Moreover, mammography is not available in most countries of SSA, and it is only available in urban centers, that made it rater costy for women living in semi-urban or rural areas to compensate for the travel and accommodation (35, 36). Another major obstacle which could also be responsible for the poor outcomes of the BC patients in Africa, is the failure to deliver the proper treatment to the patients. This is because that the treatment options for advanced stages of breast cancer are limited and restricting mainly to mastectomy, in addition to lacking other modalities including chemotherapy and/or radiotherapy facilities (37, 38). Taken together, these factors prevent many women from getting their proper medical treatment(s) for their disease. They seek for other non- medical and non- effective options such as prayer camps and herbs, and accordingly, they usually present with advanced high grade and advanced stage tumors (37). Based on the previous data we can conclude that, breast cancer is the major health problem threatening African women, owing to poverty, social and cultural barriers, as well as limited diagnostic and treatment facilities. Black et al. (30), suggested in their study that increasing public awareness for breast self-examination and clinical breast examination (CBE) could help, at least partially, in down staging of BC in the African females. This has also been supported by the relatively recent study of Dos Santos et al. (39), who reported in their study, which was done in Sudan and Tanzania, that training health workers for CBE together with awareness campaigns can effectively improve the patients’ outcomes.

## Uterine Cervical Cancer

carcinoma of the cervix uteri is among the most preventable malignancies worldwide (40), however it remains the first leading cause of cancer deaths in African women [(2), **Figure 3** **]**. Human papillomavirus (HPV) types 16 and 18 are the most common etiological factors for the pathogenesis of cervical cancer in Africa (42). The reported prevalence rate of HPV was 97.0% in Malawi (43), 92.1% in South Africa (44), 90.7% in Ibadan Nigeria (45), and 69.8% in Maiduguri and Nigeria (42). In fact, the HPV infection is usually cleared in the immunocompetent women (46). However, in women with underlying human immuno-deficiency virus (HIV) infection; as a common situation in Africa, there is an increasing risk of developing cancer cervix rather than in women without HIV infection, with the annual detection rates are 1.4 *versus* 0.4 per 100 persons per year; respectively (47–49). It was reported by de Martel et al. (50), that SSA had the highest age standardized incidence rate (ASIR) of HPV attributable cancer all over the world (ASIR 19.3 cases per 100,000 person/years). A recent meta-analysis study performed by Drolet et al. (51), including midline studies published between February 1, 2014, and October 11, 2018, reported that nearly two thirds of all cervical cancers cases caused by HPV16 and HPV18 could be prevented with the currently available HPV vaccines. At the same time, Cervical screening programs either with cytology, HPV testing, or both could prevent most of the remainder of cases especially in developed countries. However, in Africa it is rather challenged by many factors including limited resources, lack of knowledge about the cervical cancer and unavailability of screening centers (52, 53). It was estimated that the overall cervical cancer screening in Ethiopia was 0.8% according to the ICO Information Centre on HPV and Cancer 2017 (54). Similarly, it was reported to be 1% in another study done by Getachew et al. (52). All these factors contributed to inefficient early detection and consequently later diagnosis and poorer survival rates.

**Figure 3:** Regional status of incidence and mortality due to uterine cervical cancer (41).

## Hepatocellular Carcinoma

Hepatocellular carcinoma (HCC) is the third leading cause of cancer related death in Africa, and a major health problem all over the world (1). It was recorded that 80% of HCC cases occurred in the SSA and eastern Asia according to Cancer Today, which is an international agency for research and cancer (24). The prevalence of HCC is heterogeneous because it has variable risk factors, since hepatitis B (HBV) and aflatoxin exposure are the major risk factors for HCC in SSA, whereas hepatitis C (HCV) is the major risk factor for HCC in USA, Europe, and Japan (55). In a large, retrospective observational study done by Yang et al. (56), which included 2,566 patients who were treated in 21 tertiary referral centers from different countries in Africa, they observed that the African patients presented with HCC were at a younger age (median of 45 years), with advanced disease stage, severe liver dysfunction and poor performance status. Additionally, Mak et al. (57), reported that the mortality rate of HCC black African patients is higher than that in white patients. Many studies had addressed this disparity between the black and the white population, among those are Ladep et al. (58), who concluded that this disparity might be due to different biological and etiological risk factors that should be urgently identified, as those patients represent high-risk group patients who need a prompt effective treatment. Other studies attributed this poor outcome to the absence of comprehensive surveillance programs for HCC, inaccessible expert medical care, socioeconomic and sociocultural factors that affect treatment decision making (59, 60). In addition to the previously mentioned etiological factors, it is clear that the HIV epidemic has had a major demographic and health impact on the black African population, which also should be assessed (57).

## Lung Cancer

Lung cancer remains the first leading cause of cancer- related deaths in the United States (1), with the highest lung cancer mortality rate being detected in the African-American population (61, 62). Indeed, there were a conflicting data regarding the racial disparity of the prevalence and outcome of patients with lung cancer. Many studies reported a significantly lower frequencies of *EGFR* mutations in black compared white patients (63, 64). However, other groups failed to find any significant association between *EGFR* mutations and patients’ races (65, 66). An important study done by Campbell et al. (67), who performed genomic sequencing for a panel of 504 cancer genes in lung cancer tissue specimens obtained from 245 black patients compared to 264 white patients. Based on the data of their study, they concluded that there was no significant difference regarding mutational frequencies and copy number changes between the black and white patients. Also, there was no significant difference in the genetic alterations of the receptor *tyrosine kinase/Ras/Raf* pathway including *EGFR* and *KRAS*. Additionally, Mitchell et al. (68), reported no significant association between lung cancer survival and ethnic variations especially in West African ancestry. These data were confirmed by previous studies suggested that genetic ancestry did not adversely contribute to lung cancer risk or survival (69, 70). Therefore, some investigators suggested that other factors including socioeconomic, environmental or cultural variables could explain these disparities (68, 69).

Consistent with these results, Murphy et al. (71), concluded that African Americans consumed greater amounts of nicotine per cigarette compared to other American ancestry groups. This was measured by the urinary total nicotine equivalents (TNE), which is a more objective measure of smoking intensity than the number of cigarettes per day (CPD). Accordingly, TNE is correlated with the uptake of the well-known tobacco carcinogens such as *nitrosamine 4-(methylnitrosamino)-1-(3-pyridyl)-1-butanol* (NNAL) and polycyclic aromatic hydrocarbons (72). Therefore, it seems that, exomic mutations does not contribute to the observed racial disparities between black and white populations regarding lung cancer development and outcome. However, further investigations are suggested into other genomic variations such as mutations in noncoding regions and epigenetic changes, or assessment of other socioeconomic factors including smoking behavior and access to health care facilities (67).

Based on our previous discussion, we can conclude that cancer is a major public health problem in Africa, with increased incidence, financial toxicities and mortality (**Figures 4**, **5**). Racial disparities seem to played an important role for the increasing incidence and prevalence of many cancers including prostate and breast cancers which are genetically more common in black patients rather than in white population. However, the increased incidence of other cancer types including lung, hepatocellular and uterine cervical cancers could be attributed to many factors other than racial disparities. Actually, Africa is challenged by many problems including mainly the prevalence of oncogenic viruses such as *HIV* for non-Hodgkin lymphoma, *HHV-8* for Kaposi sarcoma, *HPV* for cervical cancer, *HBV* and *HCV* for HCC. Other factors including limited screening programs as PAS, TURS for prostate cancer, and mammography for breast cancer. Also included is poor implementation of *HPV* vaccines as for uterine cervical cancer and *HBV* for HCC. Moreover, African patients were challenged by poor economic circumstances, low life standard, inaccessible medical care and poor medical services. All these factors together with the racial disparities contributed to increased cancer incidence and mortality among African patients. Therefore, identifying the underlying aetiological causes for increased cancer death in Africans will contribute to better modalities for screening, diagnosis, treatment and prevention.

**Figure 4:** The most common **(A)** cancer cases, **(B)** cancer deaths in Sub-Saharan Africa, both sexes combined, 2018 (3). Reproduced from “The Cancer Atlas,” canceratlas.cancer.org (73).

**Figure 5:** Incidence and mortality rates in selected countries in Sub-Saharan Africa, 2018 (3). Reproduced from “The Cancer Atlas,” canceratlas.cancer.org (73).

## Author Contributions

AB: revised the manuscript. MA: collecting data and writing the manuscript. A-RZ: directing the work and revised the manuscript. All authors contributed to the article and approved the submitted version.

## Conflict of Interest

The authors declare that the research was conducted in the absence of any commercial or financial relationships that could be construed as a potential conflict of interest.
